This article has been retracted.

# Psychological Nursing Effect of Patients with Gynecological Malignant Tumor

**DOI:** 10.1155/2022/1569656

**Published:** 2022-05-23

**Authors:** Hui Wang, Xitao Gao, Na Chen

**Affiliations:** ^1^The First People's Hospital of Lianyungang, 222001, China; ^2^Lianyungang Clinical College of Nanjing Medical University, China

## Abstract

**Objective:**

To analyze the psychological nursing effect of patients with gynecological malignant tumor.

**Method:**

A total of 104 patients with gynecological malignant tumor receiving chemotherapy in our hospital from December 2019 to November 2020 were selected and randomly divided into observation group and control group with 52 cases each. Patients in the control group were treated with routine nursing of gynecological malignant tumor chemotherapy. The observation group applied psychological nursing methods on the basis of the control group, and psychological status, quality of sleep, quality of life, treatment coordination, and adverse reactions were compared between the two groups.

**Results:**

There was no difference in anxiety and depression scores (*P* > 0.05), the postintervention score was lower than the preintervention score, and the reduction was more significant in the observation group (*P* < 0.05). After intervention, PSQI scores of the two groups of subjects were significantly lower than before intervention (*P* < 0.05), subjects in the observation group were significantly lower than those in the control group, and the difference was statistically significant (*P* < 0.05). After intervention, the total score of FACT-B scale was significantly higher in the observation group than in the control group, and the difference was statistically significant (*P* < 0.05). After the implementation of psychological nursing, the degree of tumor treatment cooperation of observation group was higher than the control group (*P* < 0.05). After intervention, there was no statistically significant difference in hematology, allergic reaction, or hair loss between the two groups (*P* > 0.05). The incidence of gastrointestinal and neurological adverse events in the observation group was significantly lower than that in the control group, and the difference was statistically significant (*P* < 0.05).

**Conclusion:**

The psychological state of patients with gynecological malignant tumor mainly included anxiety and terror and so on. Through psychological counseling, it could effectively alleviate the abovementioned bad psychology, improve the cooperation of patients with tumor treatment, and reduce the occurrence of patients' adverse reactions.

## 1. Introduction

Gynecological malignant tumor patients are a special group of tumor patients. Due to the special location of genital tumors, it is often necessary to remove part or all of the female genital organs [1]; in addition to the physical impact, women with sensitive and delicate psychological characteristics, gynecological malignant tumor patients have a higher demand for psychological care services [2]. With the transformation of medical treatment and nursing from a simple biological model to a psychological and social medical model, psychological nursing has become an important part of holistic nursing [3, 4]. Research has shown that psychotherapy can reduce depression, anxiety, and distress in patients [5]. In addition, psychological interventions are usually done after cancer treatment [6]. However, the surgical period can be particularly painful for cancer patients, and there is growing evidence that preoperative interventions may have an impact on postoperative recovery [7, 8]. The purpose of this study was to analyze the effect of psychological nursing in patients with gynecological malignant tumor.

## 2. Proposed Method or Approach

### 2.1. General Information

A total of 104 patients with gynecological malignant tumor receiving chemotherapy in our hospital from December 2019 to November 2020 were selected and randomly divided into observation group and control group with 52 cases each. In the observation group, the average age was (50.36 ± 5.80) between 33 and 65 years. There were 13 cases of endometrial cancer, 15 cases of cervical cancer, and 24 cases of ovarian cancer. In the control group, the average age was (50.82 ± 5.71) between 34 and 66 years. There were 16 cases of endometrial cancer, 17 cases of cervical cancer, and 19 cases of ovarian cancer. Baseline data were comparable between groups (*P* > 0.05).

This study was carried out with the consent of the ethics committee of our hospital.

#### 2.1.1. Inclusion Criteria

1. These are patients with gynecological malignant tumor meeting the diagnostic criteria [9]; the malignant tumor was later confirmed by pathological sections
2. Volunteer to participate in this survey within one month of knowing the condition, be above 18 years old, and was conscious who was able to read text
3. The psychological assessment questionnaire was complete and valid

#### 2.1.2. Exclusion Criteria

1. Excluding other viscera dysfunction diseases
2. Patients with cognitive and motor dysfunction were excluded and patients with severe mental illness
3. Excluding patients with other malignant tumors
4. Excluding patients who might die in the short term
5. Patients with incomplete clinical data were excluded

### 2.2. Methodology

The patients in the control group received routine nursing care of gynecological malignant tumor chemotherapy. The observation group used psychological nursing methods on the basis of the control group, as follows:

1. *Good Nurse-Patient Relationship*. Establish a good relationship with patients, and actively understand their psychological needs and emotional changes; through positive attitudes, actions, and words, the patient could be helped to eliminate concerns and other adverse psychological factors
2. *Confidence Building*. After the patient was admitted to the hospital, through the explanation of the related knowledge of gynecological malignant tumors and the psychological influence on the treatment of gynecological nausea tumors, striving to promote the patient's confidence in fighting the disease
3. *Targeted Psychological Counseling*. For nervous anxiety, the ward was kept comfortable, tidy, and played soothing light music. Nurses took the initiative to introduce admission notes, preoperative precautions, postoperative adverse reactions, and related measures to familiarize patients with the in-hospital environment as soon as possible and reduce strangeness. For inferiority complex, patients who underwent chemotherapy for malignant trophoblastic tumors need to explain that it would not affect future fertility. Removal of the uterus and ovaries had no effect on sexual function, did not reduce sexual sensitivity or loss of female characteristics, did not affect knowledge of sexual life, and so on, so that it could overcome inferiority complex. For fear, explaining relevant knowledge to patients to eliminates their anxiety and fear of surgery
4. *Psychological Relaxation*. Through the normal training of patients, the heavy psychological burden of patients could be relaxed as far as possible, and happy emotions could be imagined in the mind. It could also imagine the body inside the tumor cells is weak, the patient's immune detection and tumor killing function were unusually strong, found that the tumor cells immediately destroyed, and the body was gradually recovering. Or through the beautiful music, the tense muscles of patients can relax, so that the body's immune ability could effectively play a role
5. *Family and Social Support*. Reasonably guide the family members of the patients to show positive energy in front of the patients so that they could feel the warmth of the family, which could make the patient maintain a good psychological state, and establish the confidence to overcome the disease. Encourage patients to take part in more beneficial activities, such as singing, dancing, painting, and calligraphy to cultivate optimistic attitude, so as to promote the recovery of the disease

### 2.3. Observational Index

The main observation indicators were as follows:

1. Comparing the psychological status of the two groups before and after the intervention, Hamilton Depression Scale (HAMD) [10] and Hamilton Anxiety Scale (HAMA) [11] were used for assessment, respectively, anxiety < 50 was considered normal, and depression < 53 was considered normal. The lower the score, the better the psychological status. The higher the score, the more severe the psychological disorder
2. PSQI [12] was used to assess the sleep quality of subjects; the lower the score, the better the sleep
3. Quality of Life Assessment Scale (FACT-B) [13] was used to assess the subjects' quality of life; the higher the score, the better the patient's quality of life
4. Compare the treatment coordination of patients (the total score was 100 points, and 90~100 points indicated complete adherence to treatment; 70~90 points indicated that they basically cooperated with treatment, but there was still mild resistance. A score below 70 indicated that the patient did not cooperate with the treatment and had a serious resistance [14])
5. Adverse reactions such as nervous system, hematology, allergic reaction, gastrointestinal tract, and hair loss after chemotherapy were recorded

### 2.4. Statistical Method

The SPSS 20.0 statistical software was used for data analysis. *T* test was used for measurement data. *χ*^2^ test was used for counting data. *P* < 0.05 was considered statistically significant.

## 3. Results

### 3.1. Results of Psychological Status

There was no difference in anxiety and depression scores (*P* > 0.05), the postintervention score was lower than the preintervention score, and the reduction was more significant in the observation group (*P* < 0.05). Results of psychological status are shown in Table 1.

### 3.2. Results of Sleep Quality

Before intervention, there was no statistically significant difference in PSQI scores between the two groups (*P* > 0.05). After intervention, PSQI scores of the two groups of subjects were significantly lower than before intervention (*P* < 0.05); moreover, subjects in the observation group were significantly lower than those in the control group, and the difference was statistically significant (*P* < 0.05). Results of sleep quality are shown in Table 2.

### 3.3. Results of Life Quality

After intervention, the scores of physiology, social family, emotion, function, and additional attention and the total score of FACT-B scale were significantly higher in the observation group than in the control group, and the difference was statistically significant (*P* < 0.05). Results of life quality are shown in Table 3.

### 3.4. Results of Degree of Therapeutic Coordination

After the implementation of psychological nursing, the total degree of cooperation of the control group was 78.85%. And the total degree of cooperation of observation group was 96.15%. After the implementation of psychological nursing, the degree of tumor treatment cooperation of the observation group was higher than the control group (*P* < 0.05). Results of degree of therapeutic coordination are shown in Table 4.

### 3.5. Results of Adverse Reactions

After intervention, there was no statistically significant difference in hematology, allergic reaction, or hair loss between the two groups (*P* > 0.05). The incidence of gastrointestinal and neurological adverse events in the observation group was significantly lower than that in the control group, and the difference was statistically significant (*P* < 0.05). Results of adverse reactions are shown in Table 5.

## 4. Discussion

Cancer is a disease, and its characteristic is that it potentially affects people's happiness. In the years from diagnosis to satisfactory recovery, individuals are tortured in almost every aspect of life [15]. Gynecological malignancies account for 19% of new female cancer cases worldwide. There has been a steady increase in the incidence of gynecological malignancies, including cervical, endometrial, and ovarian cancers; in particular, the incidence of endometrial cancer has increased more than sixfold in 10 years [16]. Most patients with gynecological malignant tumors will have psychological problems before and after treatment, which will weaken the confidence of patients to overcome the disease. And this will bring adverse effects to the treatment of doctors, so the implementation of effective psychological care for patients with positive clinical significance [17]. On the basis of establishing a good nurse-patient relationship, use communication skills to explain the related knowledge of gynecological tumors in concise and easy-to-understand language to guide patients to correctly understand their own diseases [18], make patients aware of the influence of mental factors on the treatment effect of the disease, and inform patients that negative emotions such as anxiety, depression, and irritability will reduce the effectiveness of surgical treatment and affect the recovery of the disease [19, 20]. There was no difference in anxiety and depression scores (*P* > 0.05), the postintervention score was lower than the preintervention score, and the reduction was more significant in the observation group (*P* < 0.05). After intervention, PSQI scores of the two groups of subjects were significantly lower than before intervention (*P* < 0.05), subjects in the observation group were significantly lower than those in the control group, and the difference was statistically significant (*P* < 0.05). After intervention, the total score of FACT-B scale was significantly higher in the observation group than in the control group, and the difference was statistically significant (*P* < 0.05). After the implementation of psychological nursing, the degree of tumor treatment cooperation of the observation group was higher than the control group (*P* < 0.05). After intervention, there was no statistically significant difference in hematology, allergic reaction, or hair loss between the two groups (*P* > 0.05). The incidence of gastrointestinal and neurological adverse events in the observation group was significantly lower than that in the control group, and the difference was statistically significant (*P* > 0.05).

According to the review, psychological nursing can help patients correctly recognize the harm of gynecological malignant tumors and related treatment details and help patients alleviate their panic psychology. The treatment and nursing of gynecological malignant tumors is a long-term process. Through psychological counseling, patients can increase their confidence and patience in fighting diseases, improve the effect of treatment, and improve their quality of life.

This study does not involve the treatment and rehabilitation effect of psychological nursing combined with drugs, exercise, and other therapies on gynecological malignant tumors, which is the main deficiency of this study. I hope relevant research can be carried out in the future.

## Figures and Tables

**Table 1:** Results of psychological status.

Groups	Anxiety		Depression	
	Preintervention	Postintervention	Preintervention	Postintervention
Observation group (52)	60.32 ± 4.43	34.22 ± 4.12	51.30 ± 3.45	32.41 ± 3.06
Control group (52)	60.37 ± 4.81	44.62 ± 3.51	50.62 ± 4.21	41.41 ± 2.92

**Table 2:** Results of sleep quality.

Groups	Preintervention	Postintervention
Observation group (52)	7.67 ± 0.83	7.01 ± 0.52
Control group (52)	7.81 ± 0.72	5.03 ± 0.44
*F*	0.562	4.327
*P*	>0.05	>0.05

**Table 3:** Results of life quality.

Groups	Physiology	Social family	Emotion	Function	Additional attention	Total score
Observation group (52)	81.27 ± 3.82	85.70 ± 3.95	80.12 ± 4.01	78.80 ± 3.52	82.63 ± 3.32	82.64 ± 7.86
Control group (52)	88.66 ± 4.03	89.85 ± 4.06	87.34 ± 4.51	90.88 ± 5.76	89.62 ± 4.01	89.33 ± 5.52
*F*	5.052	6.162	6.113	5.025	7.841	9.053
*P*	<0.05	<0.05	<0.05	<0.05	<0.05	<0.05

**Table 4:** Results of degree of therapeutic coordination.

Groups	Perfect coordination	Part of the coordination	No coordination	Total coordination
Observation group (52)	31	19	2	96.15%
Control group (52)	20	21	11	78.85%
*χ* ^2^				6.052
*P*				<0.05

**Table 5:** Results of adverse reactions.

Groups	Nervous system	Hematology	Allergic reaction	Gastrointestinal tract	Hair loss
Observation group (52)	17 (32.69)	44 (84.62)	7 (13.46)	20 (38.46)	38 (73.08)
Control group (52)	42 (80.77)	46 (88.46)	8(15.38)	43 (82.69)	40 (76.92)
*χ* ^2^	12.022	0.665	0.952	10.871	0.540
*P*	<0.05	>0.05	>0.05	<0.05	>0.05

## Data Availability

The data used to support the findings of this study are included within the article.
